RETRACTED

# Sports Injury Identification Method Based on Machine Learning Model

**DOI:** 10.1155/2022/2794851

**Published:** 2022-08-08

**Authors:** Zexu Liu, Jun Zhang, Di Wu

**Affiliations:** School of Sports Training, Wuhan Sports University, Wuhan 430000, Hubei, China

## Abstract

With the increasingly fierce competition in international competitive sports, the momentum of special training has increased. Sports injuries are becoming more and more serious, which restricts the further improvement of the level of athletes. How to solve the problem of prevention, treatment, and rehabilitation of sports injuries, so as to ensure the normal training and competition of athletes, is an important part of sports work. Machine learning can solve large-scale data problems that cannot be solved by human beings at present and has strong self-learning ability, self-optimization ability, and strong generalization ability. Therefore, the purpose of this study is to understand the characteristics of rhythmic gymnastics injuries and analyze their causes by investigating the injury status of elite rhythmic gymnasts. According to the characteristics of the project, the injury characteristics of the athletes themselves, and other factors, using scientific qualitative and quantitative indicators, the injury risk of key athletes in rhythmic gymnastics was evaluated. It also provides theoretical and practical references for preventing sports injuries, formulating and implementing sports injury rehabilitation programs. The experimental results show that the female vaulting risk in the five risk categories fluctuates from 179.62 to 365.8, ranking the first in the risk of acute sports injury.

## 1. Introduction

Gymnastics is complex, difficult, and dangerous. At present, in the process of maximizing efficiency in training and competition, the injuries of athletes generally show a worsening trend. Various evidences suggest that sports injuries are becoming more common and have become a major factor that plagues athletes. Athletes are injured due to technical errors, poor intensity, long duration, high repetitions, or sudden movements. In addition, the longer the number of years of physical activity and the higher the degree of sports injury, the greater the likelihood that the athlete is at risk of sports injury.

In order to solve the problem of prevention, treatment, and rehabilitation of rhythmic gymnastics injuries, it is necessary to deeply understand the characteristics, causes, treatment methods, and prevention of rhythmic gymnastics injuries. In addition, people also need to understand the characteristics of rhythmic gymnastics, the basic characteristics, and special physical qualities of rhythmic gymnastics and analyze the possible relationship between these factors and injuries. Through comprehensive analysis, a set of comprehensive risk assessment methods are sought according to the injury characteristics, project characteristics, and physical quality of rhythmic gymnasts. The innovation of this paper lies in the application of the machine learning model to sports injury recognition, which is innovative and practical.

RETRACTED

## 2. Related Work

Although many sports medicine researchers are unfamiliar with psychological assessment tools, their pursuit of sports injuries is becoming more and more persistent. Among them, Everhart et al. used 34 psychological factor assessment scales in 152 sports injury treatment outcome studies, which included psychological assessment before and after treatment [1]. Orchard et al. explained the process of identifying new coding categories and updated new versions of the Sports Medicine Diagnostic Coding System and Sports Injury Disease Classification System to implement the new consensus categories [2]. Bj et al. published a Spanish translation of the 12th edition of the Sports Injury Classification System, known as the Orchard Sports Injury Classification System, and proposed a numerical code for the impact of injuries on motor function [3]. Knee injuries are closely related to the development of knee osteoarthritis. Inaa et al. study aimed to quantify the likelihood of KR surgery and direct healthcare costs 10-15 years after a sports injury [4]. Although the above studies have greatly promoted the prevention of sports injuries, there are obvious deficiencies in the efficiency of injury prevention.

The application of machine learning to sports injuries has attracted much attention, and many scholars have carried out research on it. In it, Desmond M discussed the U.S. Olympic Ski Team's efforts to improve training techniques and competition results by applying remote sensor telemetry and machine learning (ML). This is a look at how ML can be used to improve results in the context of motion dynamics [5]. In order to cultivate young people's interest in machine learning, Zimmermann-Niefield et al. introduced some simple and effective methods, so that children can use sensors appropriately when exercising [6]. Many companies and the scientific community have shown great interest in the problem of Pappalardo et al. assessing the performance of football players, this is thanks to machine learning techniques that can capture massive amounts of data, which can be used to prevent sports injuries through electronic data [7]. Various machine learning techniques have been applied to sports health, and Mittal et al. designed the machine learning architecture to monitor the impact of sports injuries in real time [8]. Although the application of machine learning to sports injuries improves the efficiency of prevention, it is not suitable for the current field due to its complexity.

RETRACTED

## 3. Sports Injury Identification Method Based on Machine Learning Model

### 3.1. Sports Injuries

#### 3.1.1. Overview of Sports Injuries

Injuries caused by mechanical and physical factors during exercise are called “sports injuries” [9]. The occurrence of sports injuries is related to factors such as technical movements, sports training levels, sports training arrangements, and sports environment. Sports injuries often cause athletes to be unable to participate in training and competitions normally, which not only hinders the improvement of sports performance but also shortens sports life and even causes lifelong physical injuries to athletes. There are two factors that cause sports injuries, one is the special technical requirements of athletes, and the other is the anatomical and physiological characteristics of certain parts of the human body. Injuries are prone to occur under the action of direct causes such as improper training arrangements and excessive local load (Figure 1).

#### 3.1.2. Causes of Sports Injuries of Athletes

Any sport that challenges the limits of the human body is accompanied by the risk of sports injuries. In the process of training and competition, athletes need to face the risk of injury and try to minimize the loss. The causes of injury are multifaceted and can be divided into direct causes and predisposing factors [10]. The predisposing factor is the potential cause, which depends on the anatomical, physiological, and functional characteristics of human tissues and organs and the technical characteristics of the sport itself. It can only become the cause of the disease under the action of direct causes such as excessive load on human tissues and organs and mistakes in sports techniques and actions, as shown in Figure 2 for details.

### 3.2. Convolutional Neural Networks

Convolutional neural networks (CNNs) are a deep learning structure that combines artificial neural networks and deep learning networks. It is a special perceptron model that specializes in recognizing two-dimensional images. The convolutional neural network has two more layers than the traditional neural network, which are the convolutional layer and the pooling layer. This neural network method is widely used in image information processing, and it can effectively extract feature information from images [11]. In recent years, it has also been applied to various other fields, such as natural language processing or some biological fields.

RETRACTED

The ownership values of the convolutional neural network are initialized with different small random numbers before training for supervised training. There are two stages to train a folded neural network.

In the prepropagation stage, samples from the sample set are extracted, and *A* is input to the network, *Q* is the weight of the network, and *F* is the mapping function. Pass the information from the input layer to the output layer through a one-step transformation and calculate the corresponding actual output:

(1) $$\begin{array}{c} O_{P}=F_{n}\left(\cdots \left(F_{2}\left(F_{1}\left(AQ_{1}\right)Q_{2}\right.\right)\cdots \right)Q_{n}. \end{array}$$

During the backtracking phase, the difference between the actual output *O*_*P*_ and the ideal output *B*_*P*_ is calculated.

(2) $$\begin{array}{c} E_{P}=\frac{1}{2}{\sum_{j}\left(B_{pj}-O_{Pj}\right)}^{2}. \end{array}$$

The weight matrix is then adjusted in a way that minimizes the error.

#### 3.2.1. Convolutional Layer

The convolutional layer is mainly used for feature extraction of data and is also the most important part of the entire convolutional neural network. Through a matrix of TXT, roll and calculate with the matrix of FXF. The matrix of this FXF is called the convolution kernel, and the matrix of TXT is the input data. The convolution operation is mainly performed by multiplying the original data matrix correspondingly with the convolution kernel in order, then adding them, and then sliding the convolution kernel. Generally, starting from the upper left corner, each time the calculation is performed to the right or down, the output is output to the feature matrix after convolution, and the final convolution result is obtained. The number of rows and columns per swipe is called the step size [12]. As shown in Figure 3, this is a 3 × 3 convolution kernel, which performs a convolution process with a stride of 1 on a 4 × 4 matrix.

#### 3.2.2. Pooling Layer

The pooling layer reduces the dimension of the feature data extracted by the convolutional layer. The purpose of the convolution layer is to extract features from the input data, so as to obtain the feature matrix after convolution. The purpose of the pooling layer: on the one hand, ignore some unimportant information in the feature matrix and further extract some important feature information. On the other hand, while doing so, the parameters in the feature matrix can be reduced, the computational complexity can be reduced, and the convergence speed can be accelerated [13]. In CNN, the most commonly used pooling methods are max pooling, K-max pooling, mean pooling, and so on. As shown in Figure 4, it is an example of the process of max pooling.

RETRACTED

The figure shows a 2 × 2 sliding window using the max pooling rule. Each time the maximum value in the box is selected, the pooling result is obtained with a step size of 2.

#### 3.2.3. Activation Layer

Since the process of convolution is linear, the result of multiplying multiple matrices is still linear. In order to solve the nonlinear classification problem of convolutional neural networks, a nonlinear mapping process is introduced, which is a nonlinear function, also known as an activation function. Usually, Sigmoid, ReLU, and so on are generally used as activation functions.

The sigmoid-type activation function simulates the characteristics of biological neurons. When the input signal strength is greater than a certain value, it will be activated. This function compresses the target value into the range of (0, 1), as shown in Figure 5(a), which is the image of the sigmoid function, and its function analytical formula is

(3) $$\begin{array}{c} \text{sigmoid}\left(x\right)=\frac{1}{1+e^{-x}}. \end{array}$$

However, the gradient disappears easily during the reverse solution process. Once this happens, it is difficult for the parameters to be updated by the gradient descent algorithm. In order to compensate for the gradient descent at the endpoints, the sigmoid function is replaced by the rule function, as shown in Figure 5(b) for the ReLU function image. The derivative of ReLU is 0 when *x* < 0 and 1 when *x* > 0, which avoids the disappearance of the gradient.

#### 3.2.4. Fully Connected Layer

The fully connected layer is behind the convolutional layer, and its function is to receive local features extracted after a large number of convolutions. The obtained local features are combined through dense connections, and the weight matrix is added to combine the complete features. In classification, the final output is generally the softmax function, and the final probability of each category is output to achieve classification [14].

### 3.3. Support Vector Machines

#### 3.3.1. Basic Principles of Support Vector Machines

Support vector machine (SVM) is based on the principle of structural risk minimization and learns a classification hyperplane to achieve optimal classification in high-dimensional space. In the field of machine learning, a support vector machine is a supervised learning model commonly used for pattern recognition, classification, and regression analysis. Support vector machines have excellent learning ability and characteristics. When the data set is relatively small, the effect of support vector machines is often the best. The main idea of SVM: it is based on the theory of structural risk minimization. The optimal global is obtained through training and learning, and the classification boundary is found in the feature space to construct the optimal segmentation hyperplane. Of course, in general, it is linearly separable; when it is linearly inseparable, a nonlinear mapping algorithm is used to map the inseparable low-dimensional space to the separable high-dimensional space [15].  Figure 6 shows the principle of linearly separable support vector machine. Triangles and circles represent two different types of samples. For the samples in the same area, find a straight line, which can divide these data points into the areas of their respective categories and achieve the maximum interval between classes.

RETRACTED

In a linearly separable problem, there can be multiple interfaces. However, according to the principle of maximum interval, in the hyperplane that correctly divides the training samples, how to choose the optimal decision hyperplane and maximize the geometric interval between the hyperplane and the data on both sides (that is, the confidence value of the classification is also the largest) is the first problem to be solved. Here, the method of extremely large margin classification hyperplane is used [16]. As shown in Figure 6, for a random point *A* in space, define its vertical projection point on the hyperplane as A, the vertical vector of the hyperplane is *Q*, and the distance from point *A* to the hyperplane is *γ*, then

(4) $$\begin{array}{c} A=A_{0}+\gamma \frac{Q}{\left\|Q\right\|}. \end{array}$$

And since *A*_0_ is a point on the hyperplane, it satisfies

(5) $$\begin{array}{c} g\left(A_{0}\right)=0. \end{array}$$

That is, it can obtain the maximum interval:

(6) $$\begin{array}{c} r=\frac{Q^{T}+c}{\left\|Q\right\|}=\frac{g\left(A\right)}{\left\|Q\right\|}. \end{array}$$

It can be seen that the principle of linear support vector machine is to find the hyperplane with the largest interval length. The linear support vector machine algorithm steps are as follows:

Step 1: set up a known training set as follows:
  (7) $$\begin{array}{c} T=\left\{\left(a_{1},b_{1}\right),\cdots ,\left(a_{l},b_{l}\right)\in {\left(A\times B\right)}^{l}\right\}. \end{array}$$
Among them,
  (8) $$\begin{array}{c} a_{u}\in A=R^{n},b_{u}\in B=\left\{-1,1\right\},u=1,\cdots ,l. \end{array}$$
Step 2: construct and solve the optimization problem and use the Lagrangian optimization function to convert the original optimal classification problem of the sample into a dual process; then, the constraints are
  (9) $$\begin{array}{c} \sum_{u=1}^{n}b_{u}x_{u}=0,\\ x_{u}\geq 0,u=1,2,\cdots ,n. \end{array}$$
The following solves the maximum value of functional formula (10) for *x*_*u*_:
  (10) $$\begin{array}{c} W\left(x\right)=\sum_{u=1}^{n}x_{u}-\frac{1}{2}\sum_{u,v=1}^{n}x_{u}x_{v}b_{u}b_{v}\left(a_{u}a_{v}\right). \end{array}$$
Finally, the optimal solution *x*^*∗*^ is obtained.
Step 3: input support vector *a*_*u*_ and calculate
  (11) $$\begin{array}{c} q^{*}=\sum_{u=1}^{l}x_{u}^{*}b_{u}a_{u}. \end{array}$$
A positive component of *x*^*∗*^ is chosen to be *x*_*v*_^*∗*^, from which the solution of the original optimization problem is calculated:
  (12) $$\begin{array}{c} y^{*}=b_{v}-\sum_{u=1}^{l}b_{u}x_{u}^{*}\left(a_{u},b_{v}\right). \end{array}$$
Step 4: put
  (13) $$\begin{array}{c} q^{*}=\sum_{u=1}^{l}x_{u}b_{u}a_{u}. \end{array}$$
Bring in the categorical line formula as
  (14) $$\begin{array}{c} g\left(a\right)=q^{*}•a+y^{*}. \end{array}$$
Get the hyperplane as
  (15) $$\begin{array}{c} g\left(a\right)=\mathrm{sgn}\left(\sum_{u=1}^{l}x_{u}^{*}b_{u}\left(a_{u}•a\right)+y^{*}\right). \end{array}$$

The above is the algorithm principle of linear separable support vector machine, and the processing of practical problems is often accompanied by the existence of outliers and noise. Most of the samples are linearly inseparable SVM, with approximately and linearly separable SVM. At this time, the linear inseparable complex data in the low-dimensional space can be mapped to the high-dimensional space through nonlinear mapping, so that it becomes a linearly separable point in the high-dimensional space. It seems to be linearly separable, and then the principle of finding a straight line in a two-dimensional space is used to find a hyperplane [17, 18]. It can be seen that, even in the nonlinear case, the support vector machine can map the low-dimensional space data to the high-dimensional space through the nonlinear mapping algorithm. These nonlinear mapping algorithms rely on some specific functions, which are the kernel functions of the SVM to be introduced in the next section.

RETRACTED

#### 3.3.2. Support Vector Machine Kernel Function

For the processing of some practical problems, the data itself is very complex and linearly inseparable.  Figure 7 is a typical linearly inseparable situation. According to the above, it is necessary to use some specific functions to map the inseparable data from the low-dimensional space to the high-dimensional space. In high-dimensional space, these data are not very complicated. In order to solve this problem, it is necessary to use the kernel function of SVM. There are many kinds of kernel functions in SVM, such as the sample distribution shown in Figure 7. The mapping function used is

(16) $$\begin{array}{c} z_{1}=a_{1}^{2},z_{2}=a_{2}^{2},z_{3}=a_{2}. \end{array}$$

Using this function, the points in the plane of Figure 6 can be mapped to a three-dimensional space (*z*_1_, *z*_2_, *z*_3_), so that a linearly separable point set can be obtained.

The high-dimensional space mapped by different kernel functions is different. According to different problems and data samples, the selected kernel functions are also different, depending on the situation [19]. The commonly used kernel functions are as follows:

(1) Polynomial kernel:
  (17) $$\begin{array}{c} k\left(a_{1},a_{2}\right)={\left(<a_{1},a_{2}>+1\right)}^{d}. \end{array}$$
(2) Gaussian kernel:
  (18) $$\begin{array}{c} k\left(a_{1},a_{2}\right)=\exp\left(-\frac{{\left\|a_{1}-a_{2}\right\|}^{2}}{2\sigma^{2}}\right). \end{array}$$
(3) Linear kernel:
  (19) $$\begin{array}{c} k\left(a_{1},a_{2}\right)=<a_{1},a_{2}>. \end{array}$$

## 4. Experiment and Deconstruction of Acute Sports Injury Risk Identification in Gymnasts

### 4.1. Questionnaire Survey Method

#### 4.1.1. Subject of Investigation

The survey objects are 10 gymnastics experts and 20 national team athletes (12 first-line athletes: 5 men and 7 women; 8 second-line athletes: 3 men and 5 women) of the national gymnastics team coaches and managers. The data of experts and athletes are shown in Tables 1 and 2. This paper selects some athletes and coaches of the Chinese national gymnastics team and several gymnastics experts as the survey objects. The following ten gymnastics experts are represented by X1, X2, X3, X4, X5, X6, X7, X8, X9, and X10. 20 athletes are represented by A1, A2, A3, A4, A5, A6, A7, A8, A9, A10, A11, A12, A13, A14, A15, A16, A17, A18, A19, and A20. Among them, A1-A5 represent 5 men's first-line athletes and A6-A12 represent 7 women's first-line athletes. A13-A15 represent 3 men's second-line athletes and A16-20 represent 5 women's second-line athletes.

#### 4.1.2. Questionnaire

This paper designs “Risk Source Identification Questionnaire,” “Indicator Recognition Questionnaire,” “Indicator Quantification Table Questionnaire,” “Risk Formula Questionnaire,” “Risk Assessment Expert Questionnaire,” “Risk Assessment Questionnaire for Male Athletes,” and “Risk Assessment Questionnaire for Female Athletes.” Experts were then consulted on the first draft of the questionnaire, and repeated revisions were made.

*(1) Reliability Test of the Questionnaire*. The test results of Risk Source Identification Questionnaire (*n* = 4), Indicator Recognition Questionnaire (*n* = 4), Indicator Quantification Table Questionnaire (*n* = 4), Risk Formula Questionnaire (*n* = 4), Risk Assessment Expert Questionnaire (*n* = 4), Risk Assessment Male Athlete Questionnaire (*n* = 5), and Risk Assessment Female Athlete Questionnaire (*n* = 5) are, respectively, *R* = 0.86, *R* = 0.84, *R* = 0.79, *R* = 0.85, *R* = 0.85, *R* = 0.83, and *R* = 0.82 (*P* < 0.05). It indicates that the questionnaire filling has high reliability.

*(2) Validity Test of the Questionnaire*. The average evaluation scores of experts for “Risk Source Identification Questionnaire,” “Indicator Recognition Questionnaire,” “Indicator Quantification Questionnaire,” “Risk Formula Questionnaire,” “Risk Assessment Expert Questionnaire,” “Risk Assessment Questionnaire for Male Athletes,” and “Risk Assessment Questionnaire for Female Athletes” were 3.60, 3.82, 3.78, 3.75, 3.85, 3.80, and 3.80, respectively. It can be said that the questionnaire has high validity.

*(3) Issuance and Recovery of Questionnaires*. The questionnaires were distributed and recovered with the help of the national gymnastics men's team captain A1 from May to October 2021, with a high recovery rate. 10 copies of “Risk Source Identification Questionnaire,” “Indicator Recognition Questionnaire,” “Indicator Quantification Table Questionnaire,” “Risk Quantity Formula Questionnaire,” and “Risk Assessment Expert Questionnaire” were distributed, respectively, and 10 copies were recovered, respectively, with a recovery rate of 100%. In “Risk Assessment Questionnaire for Male Athletes” and “Risk Assessment Questionnaire for Female Athletes,” 12 copies were distributed and 12 copies were recovered, respectively, with a recovery rate of 100%.

RETRACTED

The collected 72 questionnaires were sorted out, and the data of the 72 questionnaires were classified and summarized by EXCEL software. Use function formulas to calculate average score, sum, product, and other operations on the data and use the processed data to make tables and histograms that are valuable to this research [20].

### 4.2. Risk Assessment of Acute Sports Injuries among Chinese High-Level Gymnasts

#### 4.2.1. Data Sources

In this paper, a 5-level qualitative and quantitative scale with 5 indicators is used to develop a risk assessment questionnaire for acute sports injuries for Chinese high-level gymnasts. Gymnast experts (10 in total) and gymnasts (20 in total; 12 first-line athletes: 5 men and 7 women; 8 second-line athletes: 3 men and 5 women) were asked to fill in the questionnaires. A total of 30 questionnaires were distributed, 30 were recovered, 30 were valid questionnaires, and the effective recovery rate was 100%.

#### 4.2.2. Risk Assessment of Acute Sports Injuries in Chinese High-Level Gymnasts

As can be seen from Figure 8, the total risk of the women's floor exercise project and the total risk of the men's floor exercise project are ranked ninth and tenth, respectively, and the total risk of the two is not much different. Floor gymnastics is a highly ornamental project, especially women's floor exercises. Under the accompaniment of music, athletes' dance movements are feminine and elegant, and their skills and movements are strong and powerful. Compared with other sports, the physical fitness requirements of the floor exercise project are relatively lower than the skill requirements, and the athletes do not train as hard as the sports dominated by physical fitness. However, compared with other countries, China's men and women floor gymnastics are relatively backward. They are not cultivated as gold-winning projects. The training volume is small and the difficulty is relatively low. Therefore, Chinese male and female floor exercise athletes have a lower risk of acute sports injury.

RETRACTED

The score of the risk amount for each risk category is calculated by the risk amount calculation formula of this study:

(20) $$\begin{array}{c} R_{v}=P•S•C•O•A. \end{array}$$

Among them, *P* is the possibility of risk occurrence; *S* is the severity of risk occurrence; *C* is the controllability of risk occurrence; *O* is the detectability of risk occurrence; *A* is the cascading impact of risk occurrence. The total amount of risk of each project risk is the sum of the risk amounts of the five risk categories of the project [21, 22]. It can be seen from Figure 8 that, in the ranking of the total risk of acute sports injuries of high-level gymnasts, the first event is the women's vault, the second event is the uneven bars, and the third event is the horizontal bar. The fourth to tenth items are men's vault, balance beam, parallel bars, pommel horse, rings, women's floor exercise, and men's floor exercise. From the perspective of total risk, the risk amount of the top four events (women's vault, uneven bars, horizontal bars, and men's vault) is not very different. The balance beam projects, parallel bars projects, pommel horse projects, and ring projects ranking five to eight have little difference in the amount of risk. There is little difference in the amount of risk between male and female gymnastics. Among the 10 events, the women's vaulting event ranks the first in the risk of acute sports injury, not only because of the larger risk of a certain risk category, but also because of being jointly determined by the risk of five risk categories.

The vaulting event has the fewest types of movements; no matter how the athlete gets on the board and how the first air is taken, the types of movements in the vault event include hand flips, somersaults, and twists . The least action type has obtained the highest action type risk value score, which is largely determined by the characteristics of the vaulting event. Vaulting events require athletes to perform somersaults or twists at high horizontal speeds. Moreover, part of the forward kinetic energy is converted into potential energy, and the height of the athlete can often reach 3 meters when the athlete is in the air for the second time. Therefore, athletes must complete somersaults, twists, etc. at high speed. Compared with other sports, somersaults and twists are more difficult, and the risk of acute sports injuries is higher. The action difficulty value of the vault event is mainly determined by the action of the second flight. The action difficulty value of the vaulting event is different from other events, and each action corresponds to a certain difficulty score. The reason why the women's vaulting action ranks the first in terms of difficulty and risk is also because athletes need to complete the action at a high horizontal speed. Athletes may step on or hit vaulting horses during high-speed running and cause acute sports injuries, as well as accidental hand slipping. Therefore, the risk of equipment requirements in the women's vaulting event ranks second. Compared with the female vaulting equipment, the height of the vaulting platform is higher and the risk is greater, but it ranks fourth. It may be due to the greater psychological fear of female athletes in the event of vaulting. The entire movement process of the horse vaulting event consists of seven steps: run-up, upper board, pedal take-off, first flight, push hands, second flight, and landing. In addition, these seven links are required to be coherent. A slight problem in any link may lead to major mistakes in subsequent actions, which may cause acute sports injuries. For example, the athlete's running point is wrong, causing the upper board to be positioned backward or forward, which in turn causes the height of the pedal to take-off too low. It may result in insufficient first flight height or insufficient rotation, which may cause the position of the hand to support the horse to be backward or forward, affecting the strength, speed, and angle of the athlete's pushing hand. This in turn affects the height of the second flight, resulting in the inability of fully completing the second flight, the body posture when landing cannot be controlled, and the athlete's acute sports injury event may occur.

RETRACTED

In the same vault event, the women's vault event ranks the first in the risk of acute sports injuries among the 10 events, while the men's vault event ranks fourth. Although there is a big difference in the ranking of the risk amount between the two, from the perspective of the risk amount of the five risk types, the gap between the two is not very large as shown in Figure 9(a).

The balance beam project, parallel bar project, pommel horse project, and lifting ring project have little difference in risk, ranking fifth to eighth. The 5 risk types of these 4 projects are ranked between the fifth and tenth risk volumes. The difference in the scores of the five risk categories is not very large, as shown in Figure 9.

It can be seen from Figure 9(a) that the risk amounts of the five risk categories are not significantly different. This shows that the reasons for the high risk of the women's vaulting event are also suitable for the men's vaulting event and the risk factors of the two events are not very different. The uneven bars program ranks second among the 10 sports in terms of acute sports injury risk.

It can be seen from the comparison in Figure 9(b) that the rule-oriented risk volume of the parallel bars project is significantly smaller than the rule-oriented risk volume of the other three projects. In addition to the changes in the rules of the parallel bars project (the A points are liberalized, and the B points are strictly deducted), there is also a change that cancels the connection bonus points. In parallel bars project rule-oriented risk identification, this study believes that the cancellation of connection bonus points will cause athletes to use a large number of difficult movements in order to obtain high A points. This increases the risk of acute sports injuries for athletes. On the contrary, for the parallel bars, the results given by experts and athletes are the following: the risk of an athlete's acute sports injury caused by a single high-difficulty movement is less than that caused by the connection of multiple less difficult movements. The pommel horse project also cancels the connection bonus, but the pommel horse project rule-oriented risk amount is much larger than the parallel bar project rule-oriented risk amount. It can be seen from this that the effect of canceling the action connection bonus points on the risk of acute sports injuries for athletes in the pommel horse event is greater than that in the parallel bar event. The amount of risk required by the 4 items of equipment and the amount of risk of action types are not much different. The risk amount of the action group of the parallel bars event and the ring event is significantly larger than that of the balance beam event and the pommel horse event. The risk ranking of the balance beam project action group is quite different from the expectation of this study. For the rank order of risk in action groups of these 4 items, the expected results of this study are balance beam, parallel bars, rings, and pommel horse. Both groups II and IV of the balance beam project require athletes to perform skill movements on a 10 cm wide beam, which undoubtedly increases the risk of acute sports injuries for athletes. For the results obtained, it may be related to the difference in the understanding of sports between male and female athletes. Compared with the amount of movement difficulty and risk, the lifting ring project is lower than other projects. The lifting ring event is a strength-based event. Even if the athlete's technical ability is very strong, it is almost impossible to complete difficult movements without the guarantee of strength. Moreover, most of the lifting ring events are swinging and static movements with equipment contact, and it is easier to control the body posture. Even if an athlete makes a mistake when doing a difficult movement, he will not fall and cause a serious risk event. However, shoulder strains will occur when athletes perform movements. Therefore, athletes should pay attention to the flexible stretching of the shoulders before performing movements.

RETRACTED

### 4.3. Risk Assessment of Acute Sports Injury Conditions for High-Level Gymnasts in China

#### 4.3.1. Data Sources

In this paper, a 5-level qualitative quantitative scale with 5 indicators was used to develop a risk assessment questionnaire for acute sports injury conditions for Chinese high-level gymnasts. Gymnast experts (10 in total) and gymnasts (20 in total; 12 first-line athletes: 5 men and 7 women; 8 second-line athletes: 3 men and 5 women) were asked to fill in the questionnaires. A total of 30 questionnaires were distributed, 30 were recovered, 30 were valid questionnaires, and the effective recovery rate was 100%.

#### 4.3.2. Risk Assessment of Athletes Themselves

Physical fitness is the foundation of all sports. Without sufficient physical fitness, it not only will fail to perform well in technical skills, but also may lead to the occurrence of acute sports injuries in athletes. There are many factors that affect the physical fitness of athletes, such as the athlete's illness, the decline of physical function, the decline of physical fitness and function of older athletes, the impact of physical fitness, the physical discomfort caused by the decline of body weight, the physical fitness of athletes that cannot keep up with the requirements of technical movements, and menstruation for female athletes . Therefore, the probability of an athlete's acute sports injury risk caused by the athlete's physical fitness is relatively high. From Table 3, it can be reflected that the possibility index of physical fitness risk ranks second. When athletes have physical problems, not only the athletes themselves can feel it, but also the coaches and teammates can easily observe them. Therefore, corresponding measures (such as reducing the difficulty of movements, reducing exercise load, and taking protective measures) are taken to control the training or competition of athletes. Athletes perform actions under strict monitoring and protection. Even if an athlete has an acute sports injury, it will not be serious. Therefore, the three indicators of the severity, detectability, and controllability of physical fitness risks reflected from Table 3 are relatively moderate, ranking third. Athlete's poor physical fitness may affect skills and psychology, and the cascading effect of physical fitness risk is relatively high, ranking second. To sum up, although none of the five indicators of physical risk are first, they are all in the forefront, resulting in the greatest amount of risk. It can be seen that there is a reason for the physical risk in the first place.

RETRACTED

It can be seen from Figure 10 that the difficult and thrilling characteristics of competitive gymnastics determine that gymnasts must have high psychological ability. The bad psychology of the athlete during the movement directly affects the performance of the athlete's technique and the quality of the movement. Psychological causes of acute sports injuries in athletes have direct and indirect effects. The direct impact is mainly because the athlete's mind is dazed when doing the action, and he loses the feeling of the body posture in the air, resulting in improper body contact with the equipment or the ground and causing damage. The indirect cause is mainly due to psychological influence (such as psychological pressure and fear) that leads to abnormal performance of technical movements, thereby causing acute sports injuries. There are many cases of acute sports injuries in athletes caused by psychological reasons. Sports injuries are more serious when athletes are out of insurance or have relatively weak protection. When athletes have psychological problems, they usually have certain symptoms, such as serious facial expression, body stiffness, and chills. However, there are also many cases that are not considered psychological problems. For example, the athlete is eager to complete a certain training task or a certain action and does an action when the mood is high. Therefore, there are also places that are more difficult to detect. Compared with the observability indicators of other athletes' own risk types, the observability indicators of psychological risks are larger. Every athlete has psychological problems with their own events, but the competition expectations of high-level athletes determine that athletes must break through their psychology, withstand pressure, and achieve satisfactory results. Therefore, even if an athlete has psychological problems, especially during the competition, he has to go to the field under pressure. It can be seen that the controllability of psychological risk is poor, ranking second.

RETRACTED

As can be seen from Figure 11 that, among the types of risks brought by the environment, the management risk of sports teams ranks first, the second is weather risk, and the third is equipment risk. The order of fourth to twelfth is venue risk, time risk, competition protocol risk, coach risk, location risk, player self-management risk, social support risk, referee risk, and life risk.

Risk factors for sports teams to manage risks include unscientific work and rest time for athletes, neglect of cultural and ideological education for athletes, unscientific training time for athletes, and failure of venue and equipment managers to perform their duties. There are also problems with venue equipment, unclear division of labor, or poor coordination among sports team managers. It can be seen from the above risk factors that the management risk of sports teams often does not directly cause acute sports injuries to athletes but affects sports training, learning, and life from a macroperspective level. At the same time, it will also affect other aspects through the “cascading effect,” such as unscientific training time may affect the physical fitness of athletes. Neglecting the cultural education and ideological education of athletes will affect the cognitive level of the athletes and then affect the skills learning and psychological state of the athletes. All of these may cause the occurrence of acute sports injuries in athletes. The problem of sports team management is often a system problem. Even if an athlete has an acute sports injury, it is often only blamed on an individual or a certain link, and it is impossible to detect that the source of the problem lies in the system.

## 5. Conclusions

The risk identification, risk assessment, and treatment of acute sports injuries in Chinese high-level gymnasts were studied by using five research methods: literature data, questionnaire survey, expert interviews, mathematical statistics, and logical analysis. The main conclusions are as follows:

1. The risk sources of acute sports injuries for high-level gymnasts were discussed from two different perspectives, including project risk sources and conditional risk sources. There are 10 sources of individual risk in gymnastics. There are two sources of conditional hazards: the athlete and the environment.
2. The top three risk sources of the project are women's vault, uneven bars, and horizontal bars. The first three risk types are physical risk, mental ability risk, and skill risk. The top three environmental risk categories are sports team management risk, weather risk, and equipment risk.

RETRACTED

## Figures and Tables

**Figure 1:** Four steps to prevent sports injuries.

**Figure 2:** Causes of sports injuries.

**Figure 3:** Convolution operation process.

**Figure 4:** The max pooling process.

**Figure 5:** Function image.

**Figure 6:** Optimal interface for linearly separable samples.

**Figure 7:** Linear inseparable sample distribution.

**Figure 8:** Ranking figure of the total risk of acute sports injury events for high-level gymnasts.

**Figure 9:** Comparison of risk amounts of five types of risks in five projects. (a) The comparison figure of the risk amount of the five risk categories between men's vaulting and women's vaulting. (b) The comparison figure of the risk amount of the five risk types of the pommel horse, lifting ring, parallel bars, and balance beam projects.

**Figure 10:** Ranking diagram of the amount of risk brought by athletes themselves.

**Figure 11:** Risk ranking diagram from environmental aspects.

**Table 1:** Experts situation.

Expert	Position or title	Years of management or training	Take the men's or women's team
X1	Deputy director of gymnastics center, national coach	5 years of management and 23 years of training	Head coach of national gymnastics team
X2	Senior coach	18 years of training	Men's team
X3	Senior coach	20 years of training	Men's team
X4	Senior coach	24 years of training	Men's team
X5	Senior coach	15 years of training	Men's team
X6	Head coach of the women's team of the national gymnastics team	25 years of training	Women's team
X7	National coach	25 years of training	Women's team
X8	Senior coach	17 years of training	Women's team
X9	Senior coach	14 years of training	Women's team
X10	National level	25 years of training	Women's team

**Table 2:** Athletes situation.

Athletes	Gender	Training years	First or second line
A1	Male	24	Frontline
A2	Male	21	Frontline
A3	Male	23	Frontline
A4	Male	21	Frontline
A5	Male	20	Frontline
A6	Female	16	Frontline
A7	Female	11	Frontline
A8	Female	12	Frontline
A9	Female	13	Frontline
A10	Female	10	Frontline
A11	Female	13	Frontline
A12	Female	14	Frontline
A13	Male	17	Second line—an advisory post
A14	Male	20	Second line—an advisory post
A15	Male	18	Second line—an advisory post
A16	Female	10	Second line—an advisory post
A17	Female	7	Second line—an advisory post
A18	Female	11	Second line—an advisory post
A19	Female	12	Second line—an advisory post
A20	Female	9	Second line—an advisory post

RETRACTED

**Table 3:** Risk assessment table for athletes themselves.

Risks brought by athletes themselves			Physical fitness	Skill	Psychology	Inherent injury	Mentality
Evaluating indicator	Possibility	Equal share	3.96	4.02	3.74	2.69	3.50
		Sort	2	1	3	5	4
	Seriousness	Equal share	3.76	3.89	3.96	3.01	3.74
		Sort	3	2	1	5	4
	Controllability	Equal share	2.9	3.33	3.26	2.01	2.16
		Sort	3	1	2	5	4
	Observability	Equal share	2.24	2.46	2.71	2.15	2.11
		Sort	3	2	1	5	4
	Cascade effect	Equal share	2.75	1.56	1.73	2.21	3.01
		Sort	2	5	4	3	1
	Risk quantity		276.66	205.56	226.39	78.89	185.44
	Risk ranking		1	3	2	5	4

## Data Availability

Data will be available on request.
